# Cinobufacini Inhibits the Development of Pancreatic Cancer Cells through the TGF*β*/Smads Pathway of Pancreatic Stellate Cells

**DOI:** 10.1155/2022/3719857

**Published:** 2022-06-30

**Authors:** Quan-Wang Li, Long-Fei Ma, Chuan-Bo Liu, Jie Zhou, Bin-Ya Ma, Yao-Xue Zhuang, Ke-Rui Zhang

**Affiliations:** ^1^Department of Oncology, Dongfang Hospital, Beijing University of Chinese Medicine, Beijing, China; ^2^Basic College of Peking Union Medical College, Beijing, China; ^3^The Second Clinical Medical College of Beijing University of Chinese Medicine, Beijing, China

## Abstract

This study aimed to test cinobufacini therapeutic potential for pancreatic cancer, verify its potential molecular mechanism, and evaluate the cinobufacini impact on pancreatic cancer microenvironment. First, the effect of cinobufacini-treated pancreatic stellate cells (PSCs) supernatant on the value-added ability of pancreatic cancer (PCCs) was tested. The results show that cinobufacini can effectively reduce the ability of PSCs supernatant to promote the value-added PCCs. Further results show that cinobufacini can effectively reduce the concentration of TGF*β* in the supernatant of PSCs. Subsequently, the impact of cinobufacini on the transcription and translation levels of key genes in the TGF*β*/Smads pathway was examined. The results showed that the impact of cinobufacini on the transcription levels of Smad2, Smad3, and Smad7 was in a concentration-dependent manner, while the transcriptional activity of collagen I mRNA was decreased with the increase of cinobufacini concentration. The results of protein expression showed that cinobufacini could upregulate the expression of inhibitory protein Smad7, inhibit the phosphorylation level of p-Smad2/3, and then suppress the expression of type I collagen (collagen I). On the one hand, this study shows that cinobufacini can inhibit the promotion of PSCs on the proliferation of PCCs. On the other hand, cinobufacini can upregulate the expression of the inhibitory molecule, Smad7, through the TGF*β*/Smads pathway and reduce the phosphorylation level of p-Smad2/3, thereby inhibiting the expression of collagen I and pancreatic fibrosis. cinobufacin can inhibit the proliferation of SW1900 cells by blocking the TGF*β*/Smads pathway of pancreatic stellate cells. These results provide a clinical basis for the treatment of pancreatic cancer.

## 1. Introduction

Pancreatic ductal adenocarcinoma (PDAC) is one of the most serious cancers, with a five-year survival rate of only 8% [1, 2]. Due to the characteristics of high-density stroma, early metastasis, hypoxic microenvironment, aggressive and drug-resistant treatment, and immune escape, 80–85% of pancreatic cancer has caused local invasion and distant metastasis at the moment of first diagnosis [3]. As a result, the opportunity for surgical resection is lost, complicating the treatment of pancreatic cancer. Despite advances in surgical treatment and adjuvant chemotherapy, first-line chemotherapy drugs such as gemcitabine are still used primarily to maintain patients' quality of life. Currently, the median survival time for PDAC is only 3–6 months, which has not improved significantly over the past few decades [3]. Therefore, in recent years, the important role of pancreatic cancer microenvironment in pancreatic cancer has become a research focus and hotspot [4].

In recent years, researchers have become increasingly aware that special microenvironments play an important role in the occurrence, invasion, and metastasis of PDAC [5]. The PDAC microenvironment refers to the stromal components surrounding pancreatic cancer cells and accounts for 80%–90% of the entire tumor volume. PDAC-rich stroma regulates tumor growth and metastasis and restricts blood perfusion and immunomodulation [6]. PDAC microenvironment includes pancreatic stellate cells (PSC) microvessels, structural proteins, and soluble cytokines.

The most striking difference between pancreatic cancer and other malignancies is pancreatic fibrosis and adhesion formation. During this process, cancer cells activate and recruit relevant stromal cells (pancreatic stellate cells and immune cells) and induce the production of matrix proteins, cytokines, chemokines, etc., resulting in hypoperfusion, hypoxia, and immunity to cancer cells, and shield the special matrix environment. Simultaneously, there is an organic interaction between cancer cells and stromal cells, which together promote the occurrence, development, invasion, and metastasis of tumors [7]. PSCs are core shapers of the pancreatic pathological microenvironment. Activated PSCs can secrete cytokines to promote cancer cell proliferation and metastasis, inhibit cancer cell apoptosis, induce tumor angiogenesis, mediate distant metastasis of cancer cells, and increase the postoperative recurrence rate of pancreatic cancer.

Relevant research reports that the TGF*β*/Smads is an important pathway to promote the production of matrix by PSCs. It plays a key role in inducing and maintaining the activation, promoting proliferation, inhibiting apoptosis, promoting matrix production, enhancing exercise capacity, and promoting the migration of PSCs [8].

Traditional Chinese medicine has certain advantages in the treatment of pancreatic cancer. Previous experiments have shown that cinobufacini can inhibit tumor growth, reduce pain, and prolong the survival of cancer patients [9]. Cinobufacin is a water-soluble preparation made from the skin of Chinese giant toads. It has the function of clearing away heat and detoxifying, reducing swelling, and dispelling blood stasis [7]. Recent studies have shown that cinobufagin can inhibit the proliferation of malignant tumor cells, induce the differentiation of tumor cells, promote the apoptosis of tumor cells, and improve the immunity of the body [10]. At present, cinobufagin has been widely used in clinical practice, especially for primary liver cancer, lung cancer, esophageal cancer, and gastric cancer. However, no studies have been reported on the effects of cinobufacini on pancreatic cancer tumor microenvironment, especially PSCs via the TGF*β*/Smads pathway. Therefore, we hypothesized that cinobufacini may interfere with PSCs through the TGF*β*/Smads pathway and further affect the pancreatic cancer microenvironment, thereby inhibiting the progression of pancreatic cancer.

## 2. Results

### 2.1. Cinobufacini Inhibits the Promotion of PSCs on the Proliferation of Pancreatic Cancer Cells

PSCs can promote the formation of the tumor microenvironment, which is beneficial to the proliferation of pancreatic cancer cells. To test whether cinobufacini affects the promotion of PSCs on the proliferation of pancreatic cancer cells, we used 0 mg/ml (control group), 1.2 mg/ml, 6 mg/ml, and 30 mg/ml concentrations of cinobufacini to treat PSCs. With the increase of the concentration of cinobufacini, the effect of PSCs supernatant (without fetal bovine serum) on the proliferation of SW1900 cell line gradually weakened (Figure 1(a)). Compared with the control group, the proliferation ability of cancer cells in each group was significantly reduced (*p* < 0.01) (Figures 1(b)–1(e)).

### 2.2. Cinobufacini Inhibits Secretion of Key Growth Factors from Pancreatic Stellate Cells

PSCs can secrete many growth factors and act on themselves, thereby continuously stimulating their activation. These growth factors can inhibit cancer cell apoptosis and promote cancer cell metastasis and proliferation. Therefore, we examined the changes of key growth factors TGF*β* and PDGF-BB in the supernatant of PSCs after treatment with cinobufacini. The results showed that, in the low- and medium-dose groups, the concentration of TGF*β* in the supernatant of PSCs was not significantly different from that in the control group, but in the high-dose group, the concentration of TGF*β* was significantly lower than that in the control group (Figure 2(a)). Under the treatment of low-, medium-, and high-doses of cinobufacini, the concentration of PDGF-BB is not significantly different from that of the control (Figure 2(b)).

### 2.3. Cinobufacini Affects the Expression of Key Gene Transcription Levels of the TGF*β*/Smads Pathway in Pancreatic Stellate Cells

TGF*β* can regulate the expression of related genes through the TGF*β*/Smads pathway, thereby promoting the progress of pancreatic cancer [10]. Our results showed that cinobufacini can effectively reduce the concentration of TGF*β* in the supernatant of PSCs. Therefore, we speculated that cinobufacini can interfere with the TGF*β*/Smads pathway of PSCs to inhibit the proliferation of PCCs and thus affect the progress of pancreatic cancer. We then examined the TGF*β*/Smads pathway key gene transcription level under different doses of cinobufacini. The results showed that, after treatment with different concentrations of cinobufacini, the transcription level of each target gene changed significantly. Among them, the expression level of Smad2 gradually increased with the increase of the concentration of cinobufacini and the transcription level in the middle- and high-dose groups was significantly higher than that in the control group (*p* < 0.05) (Figure 3(a)). The change trend of Smad3 (Figure 3(b)), Smad7 (Figure 3(c)), and Smad2 is similar, and their transcription levels also increase as the treatment concentration of cinobufacini increases. But only in the high-dose group, the transcription levels of Smad3 and Smad7 were significantly higher than those of the control group (*p* < 0.05). The trend of collagen I transcription level decreased rapidly with the increase of the concentration of cinobufacini (Figure 3(d)). The expression levels in the low-, medium-, and high-dose groups were significantly higher than those of the control group (*p* < 0.05).

After treatment with cinobufacini, as the concentration of treatment increased, the protein expression of Smad2 gradually decreased, but the difference was not significant (*p* > 0.05) (Figures 4(a) and 4(f)). Compared with the control group, the protein expression of Smad3 in the high-dose cinobufacini treatment group was slightly reduced, but the difference with the control group was still not significant (Figures 4(b) and 4(f)). The phosphorylation degree of p-Smad2/3 gradually decreased with the increase of the concentration of cinobufacini and reached a very significant level in the high-dose group (Figure 4(c) and 4(f), *p* < 0.05). The protein expression level of Smad7 gradually upregulated with the increase of the concentration of cinobufacini, and the low-, medium-, and high-dose groups were significantly higher than the control group (Figures 4(d) and 4(f), *p* < 0.05). In the high-dose group, the protein expression of collagen I was significantly reduced. But the low- and medium-dose groups were not significantly different from the control group (Figures 4(e) and 4(f)).

## 3. Discussion

One of the previous studies has shown that the use of cinobufacini local perfusion to treat pancreatic cancer can effectively inhibit tumor growth and prolong the survival of patients. However, the mechanism of alleviation of pancreatic cancer is not clear, so this study specially investigated the value-added status of PCCs under cinobufacini treatment and the changes in the transcription level and protein translation level of key genes of the TGF*β*/Smads pathway of PSCs. After cinobufacini treatment, the effect of PSCs supernatant on the proliferation of PCCs gradually decreased with the increase of cinobufacini concentration. This may be because cinobufacini interfered with the cytokine secretion state of PSCs, which changed the composition of the culture supernatant to change and led to the weakening of the promotion of proliferation. As evidenced by previous studies, cinobufagin can inhibit the proliferation of human colon cancer cells sW480 induced by TGF*β*. The mechanism may be related to promoting the increased expression of B-cadherin and reducing the expression of vimentin, which is associated with the inhibition of TGF-*β*-induced epithelial-mesenchymal processes in colorectal cancer cells [10]. Studies have shown that cinobufagin reduces the expression and phosphorylation of Smad2/3 in the TGF*β*/Smad pathway, increases the expression of Smad7, and then reduces the expression of collagen IV, thereby slowing the occurrence of renal tissue fibrosis and preventing and treating diabetic nephropathy [11, 12]. Therefore, this study considers that it is also an innovation to use the concentration and signaling pathway of cinobufasin by inducing human pancreatic cancer cells to arrest in the G2/M phase to inhibit cell proliferation and yields favorable results.

PSCs are important shapers of the microenvironment of pancreatic cancer. In the pancreatic cancer microenvironment, PSCs can activate themselves by secreting growth factors and further shape the microenvironment, thereby inhibiting cancer cell apoptosis and promoting their proliferation and metastasis [11, 12]. TGF*β* is an activator of PSCs, which can promote the epithelial-mesenchymal transition of tumor cells and also promote the secretion of various collagens by PSCs. PDGF-BB can promote the proliferation of tumor cells by activating the extracellular regulatory protein kinase pathway. Therefore, we further analyzed the changes of the key growth factors TGF*β* and PDGF-BB in the supernatant of PSCs. Under the high-dose treatment with cinobufagin, the concentrations of TGF*β* were significantly reduced, indicating that cinobufacini can change the composition of the supernatant of PSCs, thereby inhibiting the proliferation of PCCs [10].

Previous studies have shown that TGF*β* can regulate gene expression through the TGF*β*-Smads pathway [5]. After the combination of TGF*β* and TGF-*β*R, phosphorylation of receptor-associated Smad protein forms the oligomer p-Smad2/3, and then the oligomer is shed from the linker protein and freed in the cytoplasm where it is further combined with Smad4 to form a heterosource multimer. This heteromultimer is a transcription factor, which can regulate the expression of a series of genes after entering the nucleus, including matrix collagen, a-SMA, MMP-3, and MMP-9, thereby activating PSCs. The activated PSC began to express smooth muscle actin (a-SMA) and desmin, showing a fibroblast phenotype. Simultaneously, the lipid droplets originally rich in vitamin A in the cytoplasm will also disappear, the proliferative ability and exercise ability are significantly enhanced, and a large amount of extracellular matrices such as type I collagen, type II collagen, fibrin, and other extracellular matrix is secreted to promote pancreatic fibrosis [6]. The secreted extracellular matrix protein accounts for 80%–90% of the entire tumor volume. It can regulate the growth and metastasis of the tumor and improve its malignancy, restrict blood perfusion, and promote the immune escape of tumor cells [6]. A large number of cytokines and chemokines have become the core shapers of the pancreatic pathological microenvironment [13, 14]. Cinobufacin can effectively reduce the concentration of TGF*β* in the supernatant of PSCs. TGF*β* can participate in the signal transduction of the MAPK pathway, and the activation of the MAPK pathway can give tumor cells a selective growth advantage. MAPK pathway is an important cell division regulation system and plays an important role in the regulation of cell proliferation, division, and apoptosis. Therefore, the supernatant of PSCs treated with cinobufagin inhibits the proliferation of pancreatic cancer PCC cells.

However, in the process of the polymerization of the Smad2/3/4 protein, it can be blocked by the inhibitory Smad protein Smad7, which can inhibit the formation of the ortho-acidified form of p-Smad2/3 protein and block the Smad2 by the combination of special domains Smad3 polymerization and phosphorylation, thereby inhibiting the formation of transcription factors [5].

In our study, we used cinobufacin to process and detect the gene transcription level and protein coding level of the key genes of TGF*β*/Smads pathway Smad2, Smad3, and Smad7 matrix collagen, collagen I. Research data show that the transcription of the Smad2, Smad3, and Smad7 genes is gradually increased by the increase of the cinobufacini concentration. However, the changes of these three genes at the translation level are different from the transcription results, which may have different regulatory mechanisms. Among them, the change trend of mRNA transcription amount of Smad7 is consistent with the corresponding protein expression result, which may be that Huachhansu can affect the transcription activity of Smad7 protein, thereby increasing its protein expression. However, the protein expression levels of Smad2 and Smad3 were not upregulated with the increase of translation level, which may be caused by the negative feedback regulation mechanism of TGF*β*/Smads-collagen pathway. As the protein expression level of collagen I decreases, PSCs enhance the transcriptional activity of the Smad2/3 protein and then increase its protein expression, thereby promoting the content of its active form p-Smad2/3/4 transcription factor in the cell and nucleus. However, the increased expression of the inhibitory protein Smad7 inhibited the polymerization and phosphorylation of Smad2 and Smad3, which led to a decrease in the content of ortho-acidified p-Smad2/3 protein, and negative feedback regulation was inhibited. It is also possible that Huachhansu can inhibit the expression and aggregation of Smad2/3 protein at the translation level, which in turn led to a decrease in the phosphorylated p-Smad2/3 protein content. It is also possible that the two mechanisms mentioned above work simultaneously. The specific mechanism still needs further study.

This study analyzed the impact of cinobufacini on key genes of the PSC's TGF*β*/Smads pathway from perspectives of transcription and translation. The results show that cinobufacini can simultaneously change the microenvironment of pancreatic cancer from both the structure (collagen I) and the environment (soluble components), making it unfavorable for the development of pancreatic cancer.

## 4. Materials and Methods

### 4.1. Cell Lines

PSCs were purchased from Sdencell Corporation. The culture medium is a special culture medium for PSCs, Stellate Cell Media (containing 2% fetal bovine serum, 1% growth factor, and 1% double antibody: penicillin 100 U/mL and streptomycin 100 ng/mL), 37°C, 5% CO_2_, and 95% air incubator. The SW1990 cell line was purchased from the National Experimental Cell Resource Sharing Platform, in DEM medium (containing 10% fetal bovine serum and 1% double antibody: penicillin 100 U/mL and streptomycin 100 pg/mL), 37°C, 5% CO_2_, and 95% air incubator culture.

### 4.2. Cell Resuscitation and Passage

The PSCs cryopreservation tube stored in liquid nitrogen was taken, quickly warmed in a 37°C water bath, and shaken quickly to make the cryopreservation solution melt within 1 min. The cryopreservation solution-cell mixture was quickly transferred to a 15 ml centrifuge tube, and 10 ml SteM complete medium was added and centrifuged at 4°C, 1000 rpm, for 5 min; then, the supernatant was discarded, 5–7 ml Stem complete medium was added and transferred to a T25 culture flask at 37°C and 5% CO_2_ for culture.

When the cells grew to 70%–90%, the cells were subcultured. 5 ml of PBS was added to each (T25) culture flask to shake and wash, the supernatant was discarded, and this operation was repeated at least twice. 1 ml 0.05% pancreatin was added to digest for 1 min at 37°C. The shrinkage and rounding of cells were observed under a microscope and there were a few fine bubbles in suspension. When it looks like snow, 5 ml of Stem complete culture solution was added to stop the digestion. A 5 ml pipette was used to gently pipette the inner wall of the culture bottle repeatedly to make the cells wash from the bottle wall as much as possible. Then, the cell suspension was transferred to a 15 ml centrifuge tube at 4°C, 1000 rpm, for 5 min, the supernatant was discarded, and an appropriate amount of SteM was added. The cells were resuspended and passaged according to the ratio of 1: 2–1: 4, and the culture flask was placed in a 37°C and 5% CO_2_ incubator.

### 4.3. Cell Seeding and Grouping

PSCs were taken in the logarithmic growth phase, a 5 × 10^4^/mL cell suspension was inoculated in a 6-well plate, 2.5 mL per well, for 24 h, then the medium was discarded, and different treatment factors were added after adherence. Cinobufavirin with Stella Cell MEDIUM basic medium were diluted to different concentrations and added to the 6-well plate. The concentration of cinobufavirin (cinobufavirin was purchased from Anhui China Resources Jinchan Pharmaceutical Co., Ltd., national pharmaceutical approval no. 234020273) was 30 mg/ml (high-dose group), 6 mg/ml (middle-dose group), 1.2 mg/ml (low-dose group), and 0 mg/ml (control group). After 48 h, the supernatant was discarded. For cell proliferation detection, the basal medium was added again to culture for 72 h. The corresponding culture medium was collected, and centrifuged, filtered, and frozen at −20°C for later use.

For RNA extraction, it was washed three times with PBS buffer solution. Trizol solution was added at 500 M/well, fully mixed to ensure the six-well plate ground evenly contact the Trizol solution, and let stand at room temperature for 5 min. Then, it was mixed by pipetting and inhaled in a 1.5 ml EP tube −80°C frozen for future use; then, it was placed on ice for protein extraction.

### 4.4. Cell Proliferation Test

SW1990 cells in the logarithmic growth phase were digested and resuspended to obtain 1 × 10^5^/mL cell suspension, inoculated in a 96-well plate, 100 *μ*L per well, for 24 h, and PSC supernatant was added after adherence (use the supernatant of PSCs containing different concentrations of cinobufacini to treat SW1900 cells) 100 *μ*L per well; after 48 hours of treatment, CCK-810 nL complete medium 90 *μ*L was added. At 5 h, the absorbance OD value of each well was measured at a wavelength of 450 mm at the microplate reader. The experiment was repeated 3 times, with the average absorbance as the cell proliferation index.

### 4.5. ELISA

The supernatant of PSCs treated with cinobufacini for 48 h was collected, and the instruction manual (Gelatins, Shanghai, China) of the ELISA kit was strictly followed to detect the levels of TGF*β* and PDGF-BB in the supernatant of PSCs.

### 4.6. Quantitative Real-Time PCR

The cell-Trizol mixture was thawed at room temperature, 500 *µ*l of phenol chloroform was added, mixed by shaking, stand for 5 minutes, and centrifuged at 14000 rpm at 4°C for 10 minutes. The supernatant was carefully aspirated into a new centrifuge tube, and 700 *µ*l isopropanol was added, mixed well, centrifuged at 12,000 rpm at 4°C for 10 minutes; then, the supernatant was discarded and washed once with 75% ethanol; the centrifugation conditions are the same as before: air dry, dissolve in 50 *µ*l DEPC-treated water, and detected by electrophoresis. Subsequently, the qualified RNA was used to prepare cDNA using the Superscript III reverse transcription kit (ABI-Invitrogen, USA). Quantitative real-time PCR was performed using the Sybr qRT-PCR mix (ABI-Invitrogen, USA), followed by 2^−ΔΔCt^ to calculate the relative expression levels of the gene of interest. The primers of the target gene were designed using Primer premier 5 software, and the primer sequences are shown in Table 1.

### 4.7. Western Blot

Cell lysates were prepared using high-efficiency RIPA tissue/cell lysis buffer (Solarbio, Beijing, China), and then the protein content was quantified using the BCA protein assay kit (Solarbio, Beijing, China). SDS-PAGE gel electrophoresis was used to separate the same amount of protein samples and then transferred to PVDF membrane on ice (Solarbio, Beijing, China). After washing three times with TBST (10 min each) (Solarbio, Beijing, China) and then using a commercial enhanced chemiluminescence (ECL) kit (Solarbio, Beijing, China) for visualization. All antibodies are from Sant Cruz company products, the antibody source is rabbit antigen, and the primary antibody ratio is 1:200; the secondary antibody is mouse-to-rabbit, and the ratio is 1:1000.

## Figures and Tables

**Figure 1:** PCC lines and proliferation index treated with different doses of cinobufacini. 0.0 mg/ml (a), 1.2 mg/ml (b), 6.0 mg/ml (c), and 30.0 mg/ml (d). (e) PCC proliferation index after treatment with different concentrations of cinobufacini. ^#^Control group, ^*∗∗*^*p* < 0.01.

**Figure 2:** Concentration of growth factors TGF*β* and PDGF-BB in PSCs supernatant. (a) Concentration of growth factors TGF*β*. (b) Concentration of growth factors PDGF-BB. ^#^Control group, ^*∗*^*p* < 0.05.

**Figure 3:** TGF*β*/Smads pathway key gene transcription level. (a) The expression level of Smads2. (b) The expression level of Smads3. (c) The expression level of Smads7. (d) The expression level of collagen I treated with different concentrations of cinobufacini. ^#^Control group, ^*∗*^*p* < 0.05.

**Figure 4:** PSC TGFp/Smads pathway protein expression relative gray value and WB experiment results. (a–e) Smad2, Smad3, p-Smad2/3, Smad7, and collagen I protein expression relative gray value after treated with different concentrations of cinobufacini. ^#^Control group, ^*∗*^*p* < 0.05.

**Table 1:** qPCR primer information.

Genes	Forward primer	Reverse primer
Actin	GACAGGATGCAGAAGGAGATTACT	TGATCCACATCTGCTGGAAGGT
Smad2	TCCAGTATTAGTGCCCCGACA	TACTCTGTGGCTCAATTCCT
Smad3	TACAGCCATTCCATCCCCGAAA	TTCATCTGGTGGTCACTGGTT
Smad7	GTTACCCCATCTTCATCAAGTCC	AAAGCCTTGATGGAGAAACCG
Collagen I	TGGTACATCAGCAAGAACCCCAA	CGAACTGGAATCCATCGGT

## Data Availability

The datasets used during the present study are available from the corresponding author upon reasonable request. All data were processed using SPSS and GraphPad software.
